This article has been retracted.

# Rehabilitation Educational Design for Children with Autism Based on the Radial Basis Function Neural Network

**DOI:** 10.1155/2021/2961546

**Published:** 2021-11-05

**Authors:** Yueer Qi, Jia-Xuan Han

**Affiliations:** ^1^Zhijiang College of Zhejiang University of Technology, Shaoxing 312030, China; ^2^Pan Tianshou College of Architecture, Arts and Design, Ningbo University, Ningbo 315211, China

## Abstract

Children with autism need appropriate educational toys to assist rehabilitation training, so as to inhibit the development of autism. Toys and related treatments for children with autism can alleviate some of the deficits of children with autism. By using toys as stimuli and various sensations obtained by children with autism or toys as a result of reinforcement, the improvement of certain capabilities expected by related therapies can be achieved through the process of stimulation and reinforcement. However, in the process of pediatrics toy development, it is difficult for toy designers to assess whether the purpose of stimulation and reinforcement can be achieved. There are many factors that affect the design of rehabilitation toys. The industry has not formed a unified design evaluation standard, and the effects of product rehabilitation training are uneven. A method based on the radial basis function (RBF) neural network was proposed in this research to study the rehabilitation design and evaluation of rehabilitation toys for children with autism. Firstly, according to the three demand indicators for the evaluation of rehabilitation training for children with autism, that is, “useful, educational, and entertaining,” the analytic network process (ANP) method was chosen as the weighting method for determining each indicator in the overall evaluation. The RBF neural network rehabilitation model for children with autism was designed and evaluated. The maximum error of the model was less than 10%. The evaluation method was objective and reasonable, so as to provide a reference for the more accurate design evaluation, purchase, and development of rehabilitation toys for children with autism.

## 1. Introduction

The symptoms of autism in infants are mainly manifested in different degrees of language barriers, communication disorders, slender interest, and rigid behavior [1]. The brain development characteristics of children with autism are characterized by extremely fast early development, which is different from that of ordinary children. From the perspective of frontal lobe development, children with autism have two different trends: first of all, there are many cells in the frontal lobe, and the cells restrict each other, and finally, the connection with other parts of the brain cells is reduced; it results from the fact that too many frontal cells are gathered in the brain, and the cells between them are squeezed, thus causing damage to normal functions. This change leads to abnormalities in attention and mirror system function [2]. The impact of these physiological differences on children with autism is mainly manifested in poor imagination and poor communication ability, accompanied by language barriers. In terms of behavior, it is mainly a rigid, repetitive cycle of certain behaviors and poor mental guessing ability. This is a clear manifestation of the difference between children with and without autism, and it will not be improved due to age [3]. The treatment goals for children with autism are to reduce the characteristics of core autism spectrum disorders, promote learning and communication, reduce maladaptive behaviors, and maximize the final functional independence of children [4].

The treatment and rehabilitation of children with autism is a long process. In addition to the treatment of doctors and parenting, toys are an important link in the rehabilitation training process of children with autism. For children with autism, toys may be an extremely common object with few points of interest, so ordinary toys cannot attract their attention, which is enough to show that there is a certain degree of defects in their cognitive ability and imagination. The Robin Nuzzolo-Gomez study found that after baseline data, toy game adjustment sessions were conducted while free game observations were conducted. After conditioning the toy, the incidence of baseline stereotypes in children with autism is higher, the styling interval is significantly shortened, and toys play an important role. Compared with the proportion of children with Down syndrome, children with autism are unable to adapt to all stimuli and their performance is more serious. Common concerns of children with autism also show obstacles [5]. Therefore, ordinary toys may not be effective and may even cause disgust in children with autism. Therefore, how to find the design needs of children with autism for rehabilitation toys and transform them into design elements of educational toys for children with autism is a problem that many studies are paying attention to at present. Diane found that peer intervention could enhance the stimulating effect of the strategy, and the improvement of social behavior of children with autism is affected by their peers. People of the same age who have never been trained have little impact. Well-trained peers have a positive impact on children with autism [6].

In the process of designing rehabilitation toys, more attention is paid to the behavioral process for children with autism. The toy is treated as an event, emphasizing the thinking ability and process of the entire event. When a toy communicates information to a child user, or when a child communicates a certain message to a toy, interaction occurs. Rachael et al. found that the highly preferred sensory stimulus items for children with autism are related to separate play, as well as the medium preference for interactive toys [7]. Leung et al. believed that the interactive toys owned by children with autism adhere to the “people-oriented” principle, aiming at the needs of children. When toys are functional, easy to use, interesting, and educational, they are more reflective. User experience in children with autism has been widely studied for this type of research [8].

Previous studies have analyzed the characteristics and needs of rehabilitation training toys for children with autism from different perspectives and also have combined the analysis of market conditions and design demands, but they have not formed a unified standard. In the process of designing rehabilitation toys for children with autism, the formation of definite design principles and evaluation indicators is difficult to guide design practice [9]. There are too many influential factors affecting the rehabilitation training products of children with autism, the focus or thinking angles of different groups are different, and there are complex links between the various factors, which are perplexing the formulation of evaluation standards for autism rehabilitation products. Based on the previous research, this study analyzes the characteristics and needs of children with autism's rehabilitation products and introduces an analytic network process (ANP) algorithm model to optimize the evaluation index for further quantitative research. In view of the huge product evaluation system, we will conduct in-depth research on the rehabilitation-related indicators of rehabilitation training toys for children with autism.

Product rehabilitation design uses psychological methods [10] to conduct a comprehensive analysis of product form and others, so as to improve product availability. The evaluation indexes involved in the rehabilitation of rehabilitation training toys for children with autism have mutual influence and feedback relationship, which is a very complicated calculation process. The general survey analysis method and the conventional analytic hierarchy process have lower evaluation accuracy, and the ANP is selected. The ANP method is an approximation algorithm with high calculation accuracy. However, due to the need for a large number of derivative calculations, the calculation efficiency is not high. Toys for children with autism have complex properties and require a lot of calculations to produce complex data tables, which have complex forms and limited calculation accuracy. Based on the actual needs of engineering, this research proposes a design method of toys for children with autism based on RBF neural network to solve the contradiction that it is difficult to balance the calculation efficiency and calculation accuracy in design and calculation under the influence of multiple factors. RBF neural network is a kind of forward network with good performance, which is suitable for multivariate function approximation. It is widely used in the fields of adaptive filtering, function approximation, pattern recognition, and nonlinear time series prediction. Kuo et al. integrated three methods of artificial neural network data envelopment method and ANP to evaluate camera manufacturers [11]. Razmi et al. integrated ANP, fuzzy theory, and nonlinear programming to select potential suppliers as long-term partners [12]. Kuo et al. integrated fuzzy mathematics and neural network to serve the design link [13]. Soltan et al. integrated data envelopment method, decision tree, artificial neural network three methods to provide designers with choices [14], and others. Based on the analysis of the needs of the ANP, a multivariable rehabilitation toy evaluation model based on the RBF neural network was established in this study, which took into account the comprehensive impact factors of product design and more accurately restored the rehabilitation needs of children with autism. It has a certain reference value to evaluate the rehabilitation design of rehabilitation toys for children with autism.

## 2. Methodology

### 2.1. Analytic Network Process (ANP)

The analytic network process (ANP) method is a decision method suitable for the nonindependent hierarchical structure proposed by Sati [15]. The problems they face are semistructured and unstructured in nature. Both methods construct matrices, utilize the relationship between certain elements of the scale method, implement feature vectors by checking for consistency, evaluate scheme selection, and adopt the scientific method. They all use a combination of qualitative and quantitative methods to conduct research and are closely related to the subjective judgment and reasoning of decision-makers. ANP is more effective than the analytic network process (AHP) in describing and analyzing the complexity of entity relationships in the objective world [16]. ANP uses the interaction between two factors as an interaction, which can more accurately explain the complex relationship in a problem. When a complex problem has the characteristics of a nonlinear network relationship, we use the ANP to analyze the problem of AHP. The evaluation process starts with the ANP model structure. The typical structure of the ANP model includes two main parts: the control layer and the network layer. The control layer contains decision goals and decision methods. The elements of each network layer are not independent, and the interaction between elements and levels is not affiliated [17]. The classic model of the network analytic method is shown in Figure 1.

(1) $$\begin{array}{c} Q_{i}=\sum_{j=1}^{n}X_{j}Y_{ij}. \end{array}$$

In the theory and algorithm of ANP, the weight of ANP is first calculated based on the interaction between the model elements. The ANP control layer is expressed as *O*_1_,…, *O*_*n*_, and the network layer has the element group *C*_1_,…, *C*_*n*_, where *C*_*i*_ has element groups *C*_1_,…, *C*_*n*_, *e*_*i*1_,…, *e*_*ni*_, *i* = 1,…, *n*, and the control layer element *o*_*s*_ (*s* = 1,…, *m*) is quasi-criteria. Taking the element *e*_*jl*_ (*j* = 1,…, *n*_*j*_) in *C*_*j*_ as the quasi-use expert scoring method, the relevant qualitative indicators in the expert group (*S* *=* (*S*_1_, *S*_2_,…, *S*_*r*_), *r* > 1) are analyzed, and the corresponding judgment moment matrix *O*^(*k*)^ is used, *k* = 1, 2,…, *r*, where *O*^(*k*)^ represents a reciprocal matrix. There is the matrix *A*^(*K*)^ = *a*_*ij*_^(*k*)^ = lg*o*^(*k*)^ = lg*o*_*ij*_^(*k*)^ (*I*, *J* = 1, 2,…, *m*). If the overall standard deviation of the expert evaluation is expressed, namely, $\sigma_{ij}=\sqrt{\left(1/r-1\right)\sum_{k-1}^{r}{\left[b_{ij}-\left(1/r\right)\sum_{k-1}^{r}b_{ij}^{\left(k\right)}\right]}^{2}}$, then *σ*_*ij*_ being less than 1, the expert group can be considered as multiple opinions. Otherwise, experts with different opinions are selected to reevaluate or ignore them until the requirements are met. If the expert opinions are unified, the arithmetic average of the expert judgment values is used as the group judgment result. Since the average matrix of *A*^(*k*)^ does not necessarily satisfy the average consistency, the quasi-optimal transfer matrix of *O* (*O*^(*k*)^ average matrix) is obtained by using the optimal transfer matrix algorithm. The processed *O*^*∗*^ = 10^*B*^ is the initial supermatrix, among them, *B*=(1/*m*)∑_*j*=1_^*m*^(*b*_*il*_ − *b*_*jl*_), and the normalized vector is obtained.

(2) $$\begin{array}{c} W_{ij}=\left[\begin{array}{cccc} w_{i1}^{\left(j1\right)} & w_{i1}^{\left(j2\right)} & \ldots & w_{i1}^{\left(jn_{j}\right)}\\ w_{i2}^{\left(j1\right)} & w_{i2}^{\left(j2\right)} & \ldots & w_{i2}^{\left(jn_{j}\right)}\\ \ldots \\ w_{{\text{in}}_{1}}^{\left(j1\right)} & w_{ii}^{\left(j2\right)} & \ldots & w_{{\text{in}}_{i}}^{\left(jn_{j}\right)} \end{array}\right], \end{array}$$

where the column vector of *W*_*ij*_ is the degree of influence of elements *e*_*i*1_,…, *e*_*ni*_, *i* = 1,…, *n*, in *C*_*i*_ on elements *e*_*i*1_,…, *e*_*ni*_, *i* = 1,…, *n*, in *C*_*j*_. If the elements in *C*_*j*_ are not affected by the elements in *C*_*i*_, then *W*_*ij*_ = 0. In this way, the supermatrix *W* under *O*_*s*_ is finally obtained. There are *m* nonnegative matrices. The subblock *W*_*ij*_ of this matrix is column-normalized, but *W* is converse. For this reason, using *O*_*s*_ as the criterion, the importance of each group of elements under *O*_*s*_ to the criterion *C*_*j*_ (*j* = 1,…, *n*) can be compared. The ordering vector component corresponding to the element group unrelated to *C*_*j*_ is zero, thereby obtaining a weighting matrix. After the supermatrix is weighted, it becomes a weighted supermatrix, and then, the limit is calculated, that is lim_*k*⟶*∞*_*w*^*k*^. When the values of each column in the supermatrix are identical, it means that the supermatrix has reached a steady state, thereby obtaining the limit relative (impact) ranking of all elements in the element set. We sort the weights of each element in the limit supermatrix, so as to find the weight vector of the alternative, and choose the best solution based on the weight value and expert evaluation. The comprehensive evaluation formula is *Q*_*i*_=∑_*j*=1_^*n*^*X*_*j*_*Y*_*ij*_, where *Q*_*i*_ is the comprehensive index in the evaluation index system, *X*_*j*_ is the index weight of the *j*th item, and *Y*_*ij*_ is the membership degree of the *i*th evaluation object in the *j*th evaluation object. The final evaluation of the results is achieved by scoring. Here, the opinions of the experts are revised and unified, and the overall standard deviation is calculated after the experts have scored the products. When the standard deviation is less than 1, the experts' opinions are considered to be more uniform. Otherwise, experts with large differences of opinion are required to rejudge or ignore their results until the requirements are met.

### 2.2. Radial Basis Function (RBF) Neural Network

The RBF neural network is a neural network structure that simulates the local adjustment of the receiving area in the human brain. It is a feedforward network with global approximation performance, with the advantages of approximating arbitrary functions, fewer samples required for training, and high approximation accuracy [18]. This neural network has 3 layers. The input layer node passes the input signal to the hidden layer. The output layer nodes are usually simple linear functions, as shown in Figure 2.

Figure 2 shows an RBF network structure with 3 layers. Among them, *X* = (*X*_1_, *X*_2_,…, *X*_*n*_), *T* ∈ *R*^*n*^ is the network input vector, w ∈ *R*^*h*^*∗*^*m*^ is the output weight matrix, *b*_0_, *b*_1_,…, *b*_*m*_ is the output unit offset, *Y* = (*Y*_1_, *Y*_2_,…, *Y*_*m*_) is the network output, and Φ_*i*_ (*∗*) is the activation function of the *i*th hidden node. The output node in the figure indicates that the output layer neuron uses a linear activation function [15]. The structural feature of the RBF network is the basis function of the hidden baseline. The radial basis function and the distance function are used as the activation function. The most commonly used basis functions are Gaussian functions:

(3) $$\begin{array}{c} \phi_{i}\left(x\right)=\exp\left[-\frac{{\left\|x-c_{i}\right\|}^{2}}{2\sigma_{i}^{2}}\right],\;i=1,2,\ldots ,h, \end{array}$$

where *x* is an *n*-dimensional input vector, and *c*_*i*_ is the center of the *i*th basis function, a vector of the same dimension as *x*. *σ*_*i*_ is the *i*th perceived variable (the parameters can be freely selected). It determines the width of the basis function around the center point. ‖*x* − *c*_*i*_‖is the norm of the vector *x* − *c*_*i*_, which usually represents the distance between *x* and *c*_*i*_, and Φ_*i*_ (*x*) has a unique maximum at *c*_*i*_; as ‖*x* − *c*_*i*_‖ increases, Φ_*i*_ (*x*) rapidly decays to zero.

## 3. Results

### 3.1. Sample Collection

The first step is to design a supervised learning neural network to obtain sample datasets, which is also a very important and key step. The acquisition of sample data includes the collection of raw data, data analysis, variable selection, and data preprocessing. Only after the above steps are processed can the neural network learning and training be more effective. The generalization ability of neural networks is also called comprehensive ability or generalization ability [19], which means a small number of samples. It is required that the selected samples have a small correlation and representativeness. Therefore, this study selects a few typical samples from high praise products to products with a poor market response. According to the principle of the degree of difference, 100 samples of rehabilitation training toys for different types of children with autism were obtained through professional manufacturers, design companies, and market surveys. The product samples range from best-selling, high-rating products to products with a poor market response. Sources of samples include the following:

1. *Manufacturer*. The best-selling, representative products are purchased from different manufacturers mainly by telephone and on-site inspections.
2. *Market*. The best-selling and well-known samples are mainly obtained through e-commerce and physical stores. These samples can be found in the product library of the manufacturer, and the information of these samples can be found through major e-commerce companies and stores.
3. *Users*. By visiting more than 20 families, parents with rehabilitation toys for children with autism were asked, the purchase of rehabilitation toys for children with autism was recorded, and samples with many users and high popularity were finally selected.

According to the 12 indexes of rehabilitation evaluation of rehabilitation training toys for children with autism, the most similar ones were removed and 50 samples were obtained. 10 more children with autism rehabilitation training toy designers were invited to use the KJ method (also known as A-type diagram or affinity diagram) [20]. Finally, 30 typical samples were obtained. We chose 25 samples as training samples and the remaining 5 samples as test samples. 13 secondary indicators of 30 samples were scored by expert scoring and questionnaire survey, and the obtained scores were averaged to obtain the original data. Based on the determined rehabilitation design evaluation indexes for the rehabilitation training toys for children with autism, each index of these samples is given a score. The total score of each sample is calculated as the initial score data. The scoring method is a combination of questionnaire scoring and expert scoring, accounting for 50% of the total score, respectively. Part of the resulting sample data is used to train the network while the others are used to verify this network.

### 3.2. Determination of Evaluation Indicators

Under the hierarchical structure, the analytic hierarchy process uses relative scales to compare the relative importance of related elements at the same level in pairs based on human experience and judgment and comprehensively plan from top to bottom for decision goals. Based on the analytic hierarchy process, ANP considers the interaction between various factors or adjacent levels and uses a “supermatrix” to conduct a comprehensive analysis of each interaction and influencing factor to obtain its mixed weight. The determination of the relative importance index (scale) of each factor in ANP is basically consistent with that of AHP, which is obtained through questionnaire surveys of decision-makers. According to the previous research results, a three-level evaluation index system for rehabilitation toys for children with autism has been established [21], as shown in Table 1.

In the process of introducing the RPF neural network, because the calculation process is too large, the secondary index “product rehabilitation training needs” was selected for experimental evaluation research. According to the characteristics of the rehabilitation evaluation index, the index optimization and refinement were carried out, and finally, the three-level subindicators that affected the decision-making of rehabilitation evaluation of the rehabilitation training toy for children with autism were obtained. The indicators that affect the rehabilitation evaluation of rehabilitation toy product design for children with autism include (1) usability (C9): interface (CR1), interactive mode (CR2), size and shape (CR3), color (CR4), surface decoration (CR5), tactile perception (CR6), semantic communication (CR7), and comfort (CR8); (2) educational (C10): aesthetic education (CR9), intellectual education (CR10), and heuristic (CR11); (3) entertainment (C11): experience (CR12) and gameplay (CR13). The target layer is the rehabilitation of rehabilitation toys for children with autism, the control layer is the first-level indicators C9, C10, C11, and C12, and the network layer is the second-level indicators. According to the research steps of the model established in Section 2.1 of this paper, ANP is used to determine the priority among attributes. Assuming that the rehabilitation demand indicators (CRs) are independent of each other, according to the expert survey method, a triangle intuitionistic fuzzy number is used to compare the rehabilitation demand indicators in pairs to obtain a comparison matrix, and the weight W1 of the rehabilitation demand indicator is obtained. In the case of mutual opposition, the rehabilitation demand indicators (CRs) are compared pair by pair, and the comparison matrix is obtained as shown in Table 2.

We use a triangular fuzzy comparison matrix. The normalized eigenvector W1 corresponding to the maximum eigenvalue is obtained. From Table 2, we can see that when CRs are independent of each other, the relatively important indicators are CR1 and CR4, and the importance of indicators CR3 and CR2 is relatively low. Using the above method, we can complete the other steps of the model. We can see that there is a dependency and influence relationship between various indicators. For example, there are interactions between the secondary indicators under the primary indicator usability (C9), CR1 and CR2, CR3, CR4, CR7, and CR8, interdependence and influence, CR7 and C2 educational, and CR10 entertainment. There are also interactions between the secondary indicators. Therefore, the ANP network analysis method is used to judge the relative importance weight of each evaluation index. So, we continue to use the remaining secondary indicators as the criterion for scoring. We got the weight vector of each secondary indicator, as shown in Table 3.

### 3.3. Comprehensive Evaluation Model of Rehabilitation Toy Products for Children with Autism Based on the RBF Neural Network

The 13 indexes based on interactive evaluation of baby products are compared, the index with the highest similarity is removed, and 50 samples are obtained. 10 more senior infant product designers were invited to use the KJ method (also known as the A-type diagram method or affinity diagram method). The founder of KJ law was Kawakita Jiro, a Japanese. He summed up a set of methods from years of field visits. This method is silent; through the post-it notes and pens to the team experts in various fields, everyone quietly writes down their ideas, pastes open space together to discuss, and finally explores the relationship between each idea and does classification, aiming to ensure that views of everyone can be shared and that decisions can be made democratically [20]. The basic steps are simple classification and naming for subclassification and integration; this process eliminates repeated discussions [22]. After the secondary screening, 30 typical samples were finally obtained, and 13 secondary indicators of 30 samples were scored through expert scoring and questionnaire surveys. The obtained scores were averaged to obtain the original data, as shown in Table 4.

Firstly, the qualitative evaluation indicators describing the advantages and disadvantages are transformed into quantitative indicators. This method improves the generalization ability of the RBF neural network by normalizing it. The specific method is to divide the evaluation levels into sets {very poor, poor, average, better, very good}, the corresponding quantized data set is {0.2, 0.4, 0.6, 0.8, 1}, and the values of all the indicators obtained are in the interval [0, 1]. Since the rehabilitation evaluation index of rehabilitation toys for children with autism is a benefit index, its calculation method is as follows:

(4) $$\begin{array}{c} y_{kj}=\frac{x_{kj}-\min_{1\leq j\leq m}\left(x_{kj}\right)}{\max_{1\leq j\leq m}\left(x_{kj}\right)-\min_{1\leq j\leq m}\left(x_{kj}\right)}. \end{array}$$

Among them, *x*_*kj*_ is the evaluation value of the *k*th index of the *J*th sample, *y*_*kj*_ is the value after the *k*th index of the *j*th sample is normalized, and *m* is the evaluated samples number. The network output is the comprehensive score of the sample. The final calculation method is as follows:

(5) $$\begin{array}{c} O_{j}=\sum_{k=1}^{N}Q_{k}y_{kj}. \end{array}$$

Among them, *N* is the evaluation indexes number, and *Q*_*k*_ is the index weight. We used the above method to normalize the index data in MATLAB as the input of the network, and the output of the network is the comprehensive evaluation of the sample. The number of neurons in the input layer of the neural network model is the number of indicators used for product solution evaluation and has been determined to be 13. The output layer is the value of the evaluation result, and the number of neurons is 1. The model is trained by MATLAB neural network toolbox function newrb. In 30 typical samples, the training accuracy target is set to 0.0001, the walking constant spread is 30, and the display frequency of the training process is df = 1, mapping relationship from the input layer to output layer [23]. The network achieves the training accuracy required during 23 training sessions and obtains the training results, as shown in Figure 3.

The distribution of blue and green lines in Figure 3 represents the training curve and test curve, and the red line is the test curve. The abscissa indicates the number of convergence steps, and the ordinate indicates the closeness of the training curve to the target curve, that is, the convergence error. It can be seen that after iterative calculation, the network error between the training curve and the error curve is 1.06 × 10^−4^. The abscissa of Figure 4 which is the goal of the training network is 0.0001. It is found that the error between the test sample and the verification is very small. Finally, the evaluation results of autistic rehabilitation toys based on the RBF neural network were obtained. It can be used to calculate more accurate data and can be used as a neural network model for the evaluation of rehabilitation training products for children with autism.

## 4. Discussion

After training, we used MATLAB internal program sim () command to simulate the training data to view the effect of network prediction. The last 5 samples in Table 2 are used for verification, the data of the 5 samples are input into the network model, the data evaluation score results are obtained, and the data results are compared with the initial score data of the 5 samples. Finally, the evaluation result of the rehabilitation toy based on the RBF neural network is shown in Figure 4.

In the last 5 samples, the evaluation scores are ranked from highest to lowest according to the plan number as 29, 25, 28, 30, and 26. That is, the 29th product sample has the best interactivity, and the 26th product sample has the worst interactivity. It shows that the evaluation result of the model is more accurate.

Based on the network tomography analysis method, this paper proposes an expert scoring correction model for the model algorithms related to the ANP model, aiming at the rehabilitation needs of children with autism. The ANP analysis tool is designed and implemented. Through the analysis of application examples, the classification and arrangement of autism needs are more standardized. Although the determined factor weights are somewhat subjective, the algorithm improvement or the combination of models with ANP can still provide scientific decision-making methods for decision-makers. However, in practical applications, the goals, influencing factors, plans, and associations must be determined according to the characteristics of the actual problem and the development trend. Since the basic idea of the ANP model is that a large number of comparisons are needed, it should not add too many indexes, because it will not only increase the workload of the evaluator but also easily lead to inconsistent results comparison; it will reduce the reliability of decision-making, which requires attention. In ordinary regression analysis, the multiple correlation of variables will seriously endanger parameter estimation and expand model errors. Common methods to solve the above problems are ridge regression, stepwise regression, and partial least squares regression, but they are linear regression in nature. The ANP network analysis method is used to determine the weight of each indicator in the overall evaluation; on this basis, the rehabilitation design evaluation model of autism rehabilitation training toys based on RBF neural network will be used to reduce the harm of multiple correlations on sample parameters. The maximum error of the verified model is within 10%.

The artificial neural network can simulate the cognitive process of the brain to a certain extent. Compared with the statistical method, the prediction error is smaller. However, the support vector machine based on statistical machine learning has a good ability to predict small samples. A matching learning algorithm for the revised network is described in Koh and Bhd's study [24]. It uses gradient routing in the backpropagation path. This study only studied the design requirements that affect the rehabilitation interaction direction of children with autism. The discussion is still imperfect. However, there are many input variables and the training speed is slow, which indirectly affects the overall effect of the model. The analysis of weights with ANP is a good method to solve the relationship between factors. At the same time, RBF adopts a different form known as Extreme Learning Machine (ELM) and its learning is much faster. ELM has been used for prediction for various engineering problems [25]. Therefore, ANP combined with ELM will be an important direction for further research.

## 5. Conclusion

The evaluation model of autistic rehabilitation toy based on RBF neural network has objective and reasonable evaluation results, quick and easy calculation, and high accuracy of evaluation results. At the same time, using the easy-to-remember, self-learning, and adaptive features of the RBF neural network, more objective and realistic evaluation results can be obtained after expanding the sample type. Meanwhile, the rehabilitation of the autistic rehabilitation toy product design scheme can be excellent. Inferior provides an intuitive and accurate judgment basis. Compared with traditional program evaluation methods, the use of RBF and ANP in the design and evaluation of autistic rehabilitation toy products reduces the instability of human factors and improves the stability and accuracy of evaluation results. Preliminary progress has been made in the selection of product rehabilitation indicators for experimental evaluation. The next work is to further improve the evaluation model and gradually carry out a comprehensive evaluation study for the other nine secondary indicators. The sample selection in the experimental stage is based on comprehensiveness. Future research needs to expand and deepen the classification of rehabilitation toy products for children with autism, so as to improve the practical application accuracy of the evaluation model.

## Figures and Tables

**Figure 1:** Analytic network process structure.

**Figure 2:** Radial basis function neural network structure.

**Figure 3:** The training curve of the RBF neural network will affect the design parameters of toy rehabilitation.

**Figure 4:** The training curve of the RBF neural network will affect the design parameters of toy rehabilitation.

**Table 1:** Design requirements for autistic rehabilitation training toys.

Physiological needs	Product structural strength (C1), green environmental protection (C2), safety of connected components (C3), hygienic details (C4), potential hazard control (C5)
Psychological needs	Semantic transmission security (C6), aesthetics (C7), easy to learn and maintain (C8), innovative (C8)
Rehabilitation training needs	Usability (C9), education (C10), entertainment (C11)

**Table 2:** Pairwise comparison of rehabilitation need indicators (CRs) in opposing situations.

	CR1	CR2	CR3	CR4	CR5	CR6		CR13
CR1	1	((2.1, 4.3, 4.7); 0.7, 0.2)	((3.1, 3.4, 5.0); 0.8, 0.1)	((1.1, 1.4, 2.5); 0.6, 0.3)	1/((1.1, 1.5, 2.4); 0.6, 0.3)	1/((1.0, 1.7, 2.1); 0.6, 0.3)	…	1/((2.4, 4.2, 5.4); 0.7, 0.2)
CR2	1/((2.1, 4.3, 4.7); 0.7, 0.2)	1	((0.9, 1.9, 2.3); 0.5, 0.4)	1/((4.2, 4.7, 5.1); 0.6, 0.3)	1/((2.1, 3.7, 4.8); 0.8, 0.1)	1/((2.2, 4.2, 5.5); 0.7, 0.2)	…	((3.4, 5.5, 6.7); 0.7, 0.2)
CR3	1/((3.1, 3.4, 5.0); 0.8, 0.1)	1/((0.9, 1.9, 2.3); 0.5, 0.4)	1	1/((2.4, 3.9, 4.5)0.7, 0.1)	((1.2, 2.6, 4.7); 0.7, 0.2)	1/((1.0, 1.5, 2.4); 0.6, 0.3)	…	((2.2, 4.1, 5.8); 0.7, 0.2)
CR4	1/((1.1, 1.4, 2.5); 0.6, 0.3)	((4.2, 4.7, 5.1); 0.6, 0.3)	((2.4, 3.9, 4.5); 0.7, 0.1)	1	1/((3.2, 5.5, 6.7); 0.7, 0.2)	((2.4, 4.2, 5.0); 0.7, 0.2)	…	1/((1.1, 1.6, 2.6); 0.6, 0.3)
								
CR5	((1.1, 1.5, 2.4); 0.6, 0.3)	((2.1, 3.7, 4.8); 0.8, 0.1)	1/((1.2, 2.6, 4.7); 0.7, 0.2)	((3.2, 5.5, 6.7); 0.7, 0.2)	1	((2.4, 3.5, 4.6); 0.8, 0.1)	…	1/((0.8, 1.2, 2.1); 0.8, 0.1)
CR6	((1.0, 1.7, 2.1); 0.6, 0.3)	((2.2, 4.2, 5.5); 0.7, 0.2)	((1.0, 1.5, 2.4); 0.6, 0.3)	1/((2.4, 4.2, 5.0); 0.7, 0.2)	1/((2.4, 3.5, 4.6); 0.8, 0.1)	1	…	1/((0.9, 1.4, 2.2); 0.7, 0.2)
…	…	…	…	…	…	…	1	…
CR13	((2.4, 4.2, 5.4); 0.7, 0.2)	1/((3.4, 5.5, 6.7); 0.7, 0.2)	1/((2.2, 4.1, 5.8); 0.7, 0.2)	((1.1, 1.6, 2.6); 0.6, 0.3)	((0.8, 1.2, 2.1); 0.8, 0.1)	((0.9, 1.4, 2.2); 0.7, 0.2)	…	1

**Table 3:** Column feature vector *W* based on CRs, respectively.

	CR1	CR2	CR3	CR4	CR5	CR6	…	CR13
CR1	0.2687	0.3950	0.5508	0.1797	0.2687	0.1481	…	0.1171
CR2	0.1423	0.1262	0.1397	0.5516	0.1423	0.1518	…	0.5601
CR3	0.1797	0.1665	0.3047	0.2503	0.1542	0.2338	…	0.2646
CR4	0.4199	0.2495	0.4438	0.5034	0.1506	0.2309	…	0.1371
CR5	0.3745	0.3950	0.1912	0.1272	0.1687	0.4548	…	0.2330
CR6	0.1394	0.1118	0.6062	0.1191	0.3092	0.2339	…	0.0822
…	…	…	…	…	…	…	…	…
CR13	0.0662	0.0880	0.2026	0.0751	0.4663	0.0804	…	0.5477

**Table 4:** Score results for various purposes.

	CR1	CR2	CR3	CR4	CR5	CR6	CR7	CR8	CR9	CR10	CR11	CR12	CR13	Score
1	2	5	6	8	5	2	8	2	7	6	7	8	5	71
2	8	9	5	5	2	2	5	6	8	2	4	5	7	68
3	5	3	2	3	2	1	4	8	5	5	1	8	8	55
4	6	7	5	6	5	4	1	5	1	4	8	6	4	62
5	1	2	3	8	5	7	1	4	1	5	6	4	7	54
6	2	2	8	4	5	3	1	5	6	4	5	2	5	52
7	5	8	8	8	4	6	2	2	2	8	8	1	4	66
8	4	5	5	4	5	2	5	4	5	5	5	8	7	64
9	2	2	2	5	2	5	2	5	4	6	4	5	9	53
10	8	4	4	2	5	2	8	2	8	2	5	4	5	59
11	2	2	5	9	2	4	4	3	6	4	4	2	4	51
12	9	5	6	5	4	2	5	6	5	8	5	1	2	63
13	6	6	2	1	1	1	2	8	4	5	2	8	5	51
14	3	5	8	5	5	5	5	2	5	4	4	4	4	59
15	5	2	5	1	2	2	2	4	5	6	5	2	2	43
16	1	5	2	2	8	4	5	2	4	8	2	4	8	55
17	4	2	1	8	5	2	6	5	5	5	4	5	5	57
18	5	8	4	2	2	8	2	2	6	4	5	4	2	54
19	2	4	5	1	4	6	4	5	2	2	5	6	4	50
20	4	6	2	5	2	4	2	2	5	5	5	5	5	52
21	7	6	9	2	5	2	5	2	9	6	5	8	2	68
22	7	9	7	5	1	2	2	5	8	5	4	4	4	63
23	5	3	2	2	2	5	5	4	5	4	4	2	5	48
24	2	2	5	2	4	7	2	8	8	5	4	8	2	59
25	5	5	2	2	2	8	5	5	5	8	8	2	4	61
26	8	2	2	6	1	5	2	2	8	5	5	5	5	56
27	2	4	2	3	5	6	4	4	4	4	4	6	2	50
28	2	6	5	1	2	2	5	2	5	5	8	2	4	49
29	2	2	4	2	4	2	2	2	6	6	4	4	2	42
30	8	6	7	1	5	1	8	9	5	5	5	8	5	73

## Data Availability

The datasets and codes of this research are available from the author upon request.
